# Health Care System View of Human Papilloma Virus (HPV) Vaccine Acceptability by Emirati Men

**DOI:** 10.1155/2022/8294058

**Published:** 2022-01-28

**Authors:** Suzan Al Shdefat, Shamsa Al Awar, Nawal Osman, Howaida Khair, Gehan Sallam, Hassan Elbiss

**Affiliations:** ^1^Faculty of Medicine-Jordan University of Science and Technology, King Abdulla University Hospital, UAE; ^2^Chair of Obstetrics & Gynecology Department, College of Medicine & Health Sciences (CMHS), United Arab Emirates University (UAEU), Al Ain, UAE; ^3^Obstetrics and Gynecology Department, CMHS, UAEU, Al Ain, UAE; ^4^CMHS, UAEU, Al Ain, UAE

## Abstract

This is the most frequent sexually transmitted illness on the planet, and both men and women are equally vulnerable. HPV is associated with a broad variety of female disorders, including 99 percent of all cervical cancer cases. Specifically, the goal and contributions of this study are to determine Emirati men's opinions about the HPV vaccination, specifically whether they would use it themselves or allow their female relatives to use the vaccine. To collect the primary data, a statistical cross-sectional survey was conducted. This quantitative study was conducted using primary sources of data. A questionnaire survey with a sample size of 390 participants was used to collect data from 400 individuals. Male university students in the United Arab Emirati men have a weak grasp of HPV and are averse to vaccination (Ortashi et al., 2013). The percentage of Emirati men who accept the HPV vaccination is 37%. A total of 40.3% of the respondents opted not to participate in the survey at all. Eighty-six percent of the women surveyed had heard of cervical cancer, and one-third believed that they were at risk in the future. Twenty-five percent of those surveyed said that the HPV vaccination was safe, while 26% said it was unsafe. Respondents were just 3.1 percent vaccinated, and their family members were only 87% not vaccinated.

## 1. Introduction

Males and females alike are at risk for contracting this highly contagious illness. HPV is linked to a wide range of female diseases, including 99 percent of all cervical cancer cases, which is caused by HPV. Additionally, HPV is responsible for 60–90% of vaginal malignancies as well as 39% of vulvar cancers. Men's HPV infection is to blame for 39% of all penile cancers, while HPV has been linked to 39–65% of head and neck cancers and up to 88% of anal tumors in both sexes. Reduced HPV types including HPV 6 and 11 cause genital warts in both men and women, which have a substantial impact on quality of life and sometimes need extensive treatment. There is a strong correlation between HPV infection rates among affected males and their current sexual partners; thus, they are also at risk for additional high-risk HPV variations. Despite the lack of HPV research inside the Emirates (UAE), other Arabian Gulf nations have indicated a high prevalence of 11% for females [1].

The FDA authorized the use of a trivalent HPV vaccination for men aged 9–26 years in October 2009. HPV vaccine for male genital warts and anal cancer has been authorized by the FDA and Advisory Committee on Immunization Practices, respectively. In addition, vaccination of men between the ages of 9 and 26 against HPV reduces the prevalence of genital warts, which has significant health and economic advantages. As a result, it has been claimed that male HPV vaccinations may protect their present or prospective spouses against cervical cancer as well as other HPV-related disorders [2].

An HPV vaccination programmer for females entering grades 11 and 12 was introduced by Abu Dhabi's Health Authority (HAAD) in 2008. Inside the Middle East or Arab nations, Abu Dhabi is the very first state to implement HPV vaccination inside the public sector. An intensive media effort was also launched by Health Authority Abu Dhabi (HAAD), which arranged a training and awareness campaign for health care practitioners. The media and workplaces were used to spread the word. Previous research in the United Arab Emirates has shown that there is a significant lack of information regarding cervical screening and HPV vaccination among parents and healthcare professionals. Abu Dhabi's HPV vaccination rate started out at 50% but has now risen to 80%, according to HAAD. HAAD concluded that training medical professionals and educating women about the specifics of HPV infection were the most effective ways to increase HPV vaccine uptake. Studies have revealed that the most crucial element for good sentiments regarding HPV vaccination is actually knowing about it. The HPV vaccine has not yet been approved for boys in the United Arab Emirates; however, it is predicted that the health authorities in Abu Dhabi may consider providing the vaccine for guys following the completion of school immunization and a catch-up programmer. There are no studies to our knowledge that have looked at male HPV vaccination rates in the United Arab Emirates or even the Arabian Gulf states. The purpose of this research was to determine whether or not male Emirati men inside the United Arab Emirates are aware of and accept the HPV vaccine.

There are approximately 1.9 billion Muslims in the world; with almost all Arab countries being Muslim, it has been always perceived that Muslims only practice sex through marriage as any extramarital relationship is forbidden; as such, the prevalence of any STI should be low and not warranting any preventative measures [3].

Several research on human papillomavirus (HPV) inside the Middle East-North Africa area (MENA) region found that HPV prevalence was low compared to other western nations, until lately when certain studies showed an increase in the frequency of HPV. It was found that 17.8 percent of women in Oman had HPV infection [4] while another study approximated the prevalence of high-risk human papillomavirus (HPV) between many women living in some GCC countries and found that (21 percent) tested positive for HR-HPV, which was found to be linked to the correlation among HR-HPV infection types as well as cytology results. The most common kind of infection was other non-HPV genotype 16 (HPV16)/HPV18 HR-HPV, which accounted for 63.7% of all cases. Arab women exhibited a much lower rate of HR-HPV positive in comparison to non-Arabs (31.6% vs. 16.4%). More than one-third of women living in Qatar were found to be positive for HR-HPV, followed by those living in Bahrain, the United Arab Emirates, and Saudi Arabia (14.7%) [5–12].

Estimates reveal that every year, 569,847 females are diagnosed with cervical cancer as 311,365 died from the condition. HPV infection is the most prevalent sexually transmitted infection in the world [13–15].

The third most common malignancy in women worldwide is cervical cancer. Immediately after becoming sexually active, both men and women are at risk of contracting a sexually transmitted disease (STI). Sexual transmission of HPV does not need penetrative intercourse. Gnawing on each other's private parts is a well-known method of transmission as the most frequent HPV-related illness; cervical cancer is the most common. Cervical cancers are almost always caused by HPV infection, which accounts for the vast majority of these instances [16–18].

Cervical cancer is caused by HPV in 99 percent of instances. Additionally, HPV is responsible for 60–90% of vaginal malignancies as well as 39% of vulvar tumors. Approximately to 39% of urethral malignancies are caused by HPV infection in men. HPV has been linked to 40–70% of head as well as neck cancers including up to 80% of anterior tumors in both sexes. Genital warts caused by low-risk HPV subtypes are common in both sexes and have a significant negative influence on one's quality of life. The sexual behavior in this hot region of the world is evolving rapidly in a risky manner, due to the introduction of new standards into this virgin community along with massive globalization, the wide spread use of information technology, migration, and political changes [19–21].

There are several reasons why STI prevention is so important in the Arab world, which has one of the world's youngest populations. In 2008, Abu Dhabi's Health Authority for Abu Dhabi (HAAD) incorporated HPV vaccine in its immunization programmed. Vaccination for females entering grades 11 and 12 inside the Middle East or Arab nations, Abu Dhabi is first state to implement HPV vaccination inside the public sector [22].

### 1.1. Objectives

The present study is aimed at investigating the attitude of Emirati men towards HPV vaccine, whether they will use it themselves or allow their female relatives to use it.

## 2. Material and Method

If you conceive of research as an umbrella phrase that incorporates a variety of tasks, you will be on the right track. In order to solve philosophical and practical questions, researchers use rigorous methods. According to the methodology and setting of the research, there are a variety of methodologies, including (a) descriptive analysis, which focuses on obtaining information that establishes the presence of what is being studied; (b) an evaluation and evaluation based on the review of information; (c) applicable analysis may be utilized in product, process, or policy development; and (d) foundational research is performed to fulfill scientific interest instead of for immediate practical application. There are many aspects that are not measurable and consequently cannot be estimated or interpreted quantitatively in qualitative research (e). There are much more instruments and procedures involved in quantitative research (f) than there are in qualitative research [23].

### 2.1. Study Approach and Strategies

In order to acquire the main data, a statistical cross-sectional survey was undertaken. Based on the original data, this statistical analysis was conducted. There were 390 participants in the questionnaire survey that collected data from 400 people.

### 2.2. Data Analysis

Analysis and interpretation of the acquired data were carried out using IBM SPSS. Descriptive research was used to effectively understand the study's findings [21] . Researchers often see interpretivism as a kind of qualitative analysis. This study makes use of descriptive research methods. Descriptive analytic design is used to define new information about individuals, events or behaviors, settings, or the occurrence of such events [22]. Descriptive research may be used to describe any study's findings and features [23].

### 2.3. Population

The United Arab Emirates men constitute the study's research study population.

### 2.4. Materials/Instruments

The original data was used in this quantitative study; a sample of 390 survey respondents was employed to gather data, and a questionnaire survey was used to do so [14, 24].

## 3. Results

Prevalence of the taking HPV vaccine by respondents shows 37% acceptance rate which can be seen in Table 1, 40.3% of the respondent gives refused to respond as show in Tables 1 and 2 and Figures 1 and 2.

HPV vaccine recommendation for respondents' daughters, relatives, or friends shows 46.7% yes response while 22.8% no response as given in Table 2 and Figure 2.

Table 3 and Figure 3 show the respondent attitude towards HPV vaccine which shows 21.3% response in good as it can prevent cervical cancer. 4.6% of the respondents show that vaccine is good but not safe, while good but not culturally acceptable is shown by 4.1% of the overall respondents. 1.8% of the respondents show that vaccine is not good, while bad and should not be used were responded by 1.3% of the overall respondents. 7.9% of the respondents almost show no response on the attitude towards HPV vaccine.

Table 4 shows that opinion of respondents towards HPV vaccine shows 0.3 percent response that vaccine is good as it prevents cervical cancer but not good as it is culturally unaccepted, and all of the other dimensions also responded 0.3%.

Table 5 shows that the opinion and barriers might arise in free introduction of vaccine which shows that no barrier was responded by 23.6% of the respondents. 11.3 respondents show culturally unacceptable; meanwhile, 2.1% respondents show that vaccine is religiously unacceptable; 5.4% gives their response in women usually are least concerned about their own health. 44% of the population is not aware of the situation.

Table 6 investigated the factors upon which HPV vaccine is not taken by the respondents which shows 0.3% of the population is afraid that it will not work. 0.3% of the population is not using it because of cost; 0.3 is feeling that vaccine is culturally unacceptable and due to lack of education/knowledge. 1% of the respondents are not taking it because of religiously unacceptable, while 0.3% because of side effects and decreased body immunity.

Table 7 shows the respondents' recommendations about HPV vaccine; 20.5% recommend it safe, while 22.6% respondents did not recommended it as it is not safe.

Table 8 shows the recommendations whether it is recommended by doctors which shows 9.7% yes response while 33.3% no response from the respondents.

Table 9 shows the recommendations based by family members, which shows that 1.5% of respondents were recommended by family members, while 41.5% of the respondents were not.

Table 10 shows that the recommendation by the health programs in media is investigated in Table 10, upon which respondents show 13.3 yes response, while 29.7% shows no response.

Table 11 shows recommendations by the religious authorities, which shows 41% of the respondents will not recommend even it was recommended by the religious authority while 2.1% were recommended.

Table 12 shows that recommendations by the others show that 1% of the respondents would recommend vaccine while 57.9% of the respondents will not; 13.8 of the respondents did not show the response overall.

Table 13 shows that assessment of taking the HPV vaccine by respondents shows that only 3.1% respondents have taken the vaccine while 87.4% of the respondents did not take the HPV vaccine as given in Table 13.

Table 14 shows that the assessment of either any family member of the respondents has taken the vaccine which shows that 11% of the respondent's family has taken the HPV vaccine while 69% of the respondent's family did not taken the HPV vaccine.

Table 15 shows which family members have taken the vaccine assessment. It shows that 1.8% of the daughters, cousins, nieces, sisters, and wives have taken the HPV vaccine.

Table 16 and Figure 4 show assessment of respondents' daughters even having HPV vaccine shows that 4.9% of the respondent's daughters have taken the vaccine while 36.4% of the respondent's daughters haven't taken it yet.

## 4. Discussions

We studied whether or not men in the United Arab Emirates were aware of and willing to get HPV vaccinations, as well as variables that enhanced or lowered their chance of doing so. Prevalence of the taking HPV vaccine by Emirati men shows 37% acceptance rate which also concise with the results of Mahmud et al. [24]; 40.3% of the respondents refused to response at all. HPV vaccine recommendation for respondents' daughters, relatives, or friends shows 46.7% yes response while 22.8% no response as given in the present studies while Al-Saadi et al. [21] found that 86.7 percent of the women polled had heard about cervical cancer before, and 13.0 percent of those surveyed thought they would be at risk for the condition in the future.

The research revealed that males in the United Arab Emirates were aware of and willing to get HPV vaccines, as well as factors that increased or decreased their likelihood of doing so. The prevalence of HPV vaccination among Emirati males is 37%, which is consistent with Mahmud et al.'s [24] finding that 40.3 percent of respondents did not answer at all. HPV vaccine recommendation for respondents' daughters, relatives, or friends received a 46.7 percent yes response and a 22.8 percent no response in the current studies, while discovered that 86.7 percent of women polled had heard of cervical cancer previously and 13.0 percent believed that they would be at risk for the disease in the future. Respondents' view toward HPV vaccination, which showed a 21.3 percent response rate, is favorable since it may prevent cervical cancer. 4.6 percent of respondents believe that vaccines are beneficial but not safe, while 4.1 percent believe that they are beneficial but not culturally acceptable. 1.8 percent of respondents said that vaccines are not beneficial, while 1.3 percent of respondents indicated that vaccines are harmful and should not be used. 7.9 percent of respondents almost completely lack an opinion on the HPV vaccination. Respondents' attitudes on HPV vaccine indicate that 0.3 percent believe that the vaccine is beneficial because it prevents cervical cancer but is detrimental since it is culturally unaccepted, and 0.3 percent agree on all other aspects. Opinions and hurdles may occur during the free introduction of vaccines, which demonstrates that there are no barriers, were answered to by 23.6 percent of respondents. 11.3 respondents indicate that vaccines are culturally inappropriate; yet, 2.1 percent indicate that vaccines are religiously unsuitable, and 5.4 percent indicate that women are often the least worried about their own health. 44% of the population is oblivious to the problem.

Data were obtained using a self-administered questionnaire and based on convenience sampling in our research. As a result, we decided to conduct a self-administered questionnaire in the conservative UAE community because of the cultural sensitivities of our questions. The low response rate of 71%, which is typical for self-administered surveys, might be a drawback.

The study's key strength is that it is the first to examine sexual activities, understanding of HPV, and acceptance of HPV vaccination among UAE guys. There is a lack of data on sexual activity in our environment since sexual matters are often seen as taboo.

## 5. Conclusions

For the research, it was determined whether or not males in the United Arab Emirates knew and were willing to acquire HPV vaccines and what factors influenced this decision. When it comes to getting the HPV vaccination, Emirati males had a 37% acceptance rate, which is in line with findings by Mahmud and colleagues [24], who found that 40% of respondents did not reply at all. 46.7 percent of those polled say yes, while 22.8 percent say no to the current study's HPV vaccine recommendation for their daughters, relatives, or friends. 21.3% of respondents in this survey saw the HPV vaccination, which may prevent cervical cancer, as a positive thing. 4.6% of those polled believe that vaccines are effective but dangerous, while 4.1% believe vaccines are effective but unpalatable to the culture at large, according to the results. 1.8 percent of those polled believe that vaccines are harmful, while 1.3 percent believe that vaccines are harmful and should not be used at any cost. 7.9 percent of those polled seem to have little or no opinion on the HPV vaccine. According to HPV vaccination opinion, 0.3 percent of respondents said that the vaccine is excellent since it reduces cervical cancer but not good because it is culturally unaccepted. 23.6 percent of those surveyed said that there may be some opposition to the unfettered introduction of vaccines that exhibit no restrictions. 11.3 percent of respondents said that vaccines are culturally undesirable, while 2.1 percent stated that vaccines are religiously inappropriate, and 5.4 percent stated that women are often the least worried about their own health. Over half the public does not know about it; probably another health media campaign that targets Emirati men can help introduce the vaccine and explain that men need the vaccine exactly like women do.

## Figures and Tables

**Figure 1:** Taking HPV vaccine yourself.

**Figure 2:** Recommendation HPV vaccine for daughter, relative, or friends.

**Figure 3:** Think of HPV vaccines.

**Figure 4:** Graphical representation of the responses.

**Table 1:** Prevalence of the taking HPV vaccine by respondents.

Would you consider taking HPV vaccine yourself					
		Frequency	Percent	Valid percent	Cumulative percent
Valid	No	157	40.3	40.4	40.4
	Yes	147	37.7	37.8	78.1
	No response	82	21.0	21.1	99.2
	Not applicable	3	0.8	0.8	100.0
	Total	389	99.7	100.0	
Missing	System	1	0.3		
Total		390	100.0		

**Table 2:** HPV vaccine recommendation for respondents' daughters, relatives, or friends.

Would you recommend HPV vaccine for your daughter, relative, or friends					
		Frequency	Percent	Valid percent	Cumulative percent
Valid	No	89	22.8	22.9	22.9
	Yes	182	46.7	46.8	69.7
	No response	113	29.0	29.0	98.7
	Not applicable	5	1.3	1.3	100.0
	Total	389	99.7	100.0	
Missing	System	1	0.3		
Total		390	100.0		

**Table 3:** Respondent attitude towards HPV vaccine.

What do you think of HPV vaccine					
		Frequency	Percent	Valid percent	Cumulative percent
Valid	Good as it can prevent cervical cancer	83	21.3	21.3	21.3
	Good but not safe	18	4.6	4.6	26.0
	Good but not culturally acceptable	16	4.1	4.1	30.1
	Not good	7	1.8	1.8	31.9
	Bad and should not be given at all	5	1.3	1.3	33.2
	Others	7	1.8	1.8	35.0
	Do not know	218	55.9	56.0	91.0
	No response	31	7.9	8.0	99.0
	Not applicable	4	1.0	1.0	100.0
	Total	389	99.7	100.0	
Missing	System	1	0.3		
Total		390	100.0		

**Table 4:** Opinion of respondents towards HPV vaccine.

Q203 others					
		Frequency	Percent	Valid percent	Cumulative percent
Valid		385	98.7	98.7	98.7
	Good as it prevents cervical cancer but not good as it is culturally unaccepted	1	0.3	0.3	99.0
	Good because it prevents cervical cancer but it is not culturally accepted	1	0.3	0.3	99.2
	Good but not culturally acceptable	1	0.3	0.3	99.5
	Good if it was scientifically proven and authorized	1	0.3	0.3	99.7
	I do not try it	1	0.3	0.3	100.0
	Total	390	100.0	100.0	

**Table 5:** Barriers might arise in free introduction of HPV.

In your opinion, what barriers might arise in free introduction of HPV vaccine					
		Frequency	Percent	Valid percent	Cumulative percent
Valid	No barriers	92	23.6	23.7	23.7
	Culturally unacceptable	44	11.3	11.3	35.0
	Religiously unacceptable	8	2.1	2.1	37.0
	Women usually are least concerned about their own health	21	5.4	5.4	42.4
	Others	16	4.1	4.1	46.5
	Do not know	173	44.4	44.5	91.0
	No response	30	7.7	7.7	98.7
	Not applicable	5	1.3	1.3	100.0
	Total	389	99.7	100.0	
Missing	System	1	0.3		
Total		390	100.0		

**Table 6:** Investigated the factors upon which HPV vaccine.

Q204 others					
		Frequency	Percent	Valid percent	Cumulative percent
Valid		373	95.6	95.6	95.6
	Afraid it is not working	1	0.3	0.3	95.9
	Cost	1	0.3	0.3	96.2
	Culturally unacceptable	1	0.3	0.3	96.4
	Culturally and religiously unacceptable	2	0.5	0.5	96.9
	Health issues	1	0.3	0.3	97.2
	Lack of education	1	0.3	0.3	97.4
	Lack of general knowledge of type of virus and complications	1	0.3	0.3	97.7
	Lack of knowledge	2	0.5	0.5	98.2
	Lack of knowledge of vaccine	1	0.3	0.3	98.5
	Religiously unacceptable	4	1.0	1.0	99.5
	Side effect	1	0.3	0.3	99.7
	Side effects and decrease body immunity	1	0.3	0.3	100.0
	Total	390	100.0	100.0	

**Table 7:** Respondents' recommendations about HPV vaccine.

If you recommend HPV vaccine, you would recommend it if/it is safe					
		Frequency	Percent	Valid percent	Cumulative percent
Valid	No	88	22.6	22.6	22.6
	Yes	80	20.5	20.6	43.2
	Do not know	168	43.1	43.2	86.4
	No response	47	12.1	12.1	98.5
	Not applicable	6	1.5	1.5	100.0
	Total	389	99.7	100.0	
Missing	System	1	0.3		
Total		390	100.0		

**Table 8:** The recommendations whether it is recommended by doctors.

If recommend HPV vaccine, you would recommend it if/it is recommended by doctors					
		Frequency	Percent	Valid percent	Cumulative percent
Valid	No	130	33.3	33.4	33.4
	Yes	38	9.7	9.8	43.2
	Do not know	153	39.2	39.3	82.5
	No response	57	14.6	14.7	97.2
	Not applicable	11	2.8	2.8	100.0
	Total	389	99.7	100.0	
Missing	System	1	0.3		
Total		390	100.0		

**Table 9:** The recommendations based by family members.

If recommend HPV vaccine, you would recommend it if/it is recommended by family					
		Frequency	Percent	Valid percent	Cumulative percent
Valid	No	162	41.5	41.6	41.6
	Yes	6	1.5	1.5	43.2
	Do not know	153	39.2	39.3	82.5
	No response	57	14.6	14.7	97.2
	Not applicable	11	2.8	2.8	100.0
	Total	389	99.7	100.0	
Missing	System	1	0.3		
Total		390	100.0		

**Table 10:** The recommendation by the health programs in media was investigated.

If recommend HPV vaccine, you would recommend it if/it is recommended by health programs in media					
		Frequency	Percent	Valid percent	Cumulative percent
Valid	No	116	29.7	29.8	29.8
	Yes	52	13.3	13.4	43.2
	Do not know	153	39.2	39.3	82.5
	No response	57	14.6	14.7	97.2
	Not applicable	11	2.8	2.8	100.0
	Total	389	99.7	100.0	
Missing	System	1	0.3		
Total		390	100.0		

**Table 11:** Recommendations by the religious authorities.

If recommend HPV vaccine, you would recommend it if/it is recommended by religious authority					
		Frequency	Percent	Valid percent	Cumulative percent
Valid	No	160	41.0	41.1	41.1
	Yes	8	2.1	2.1	43.2
	Do not know	153	39.2	39.3	82.5
	No response	57	14.6	14.7	97.2
	Not applicable	11	2.8	2.8	100.0
	Total	389	99.7	100.0	
Missing	System	1	0.3		
Total		390	100.0		

**Table 12:** Recommendations by the others.

If recommend HPV vaccine, you would recommend it if/others					
		Frequency	Percent	Valid percent	Cumulative percent
Valid	No	226	57.9	58.1	58.1
	Yes	4	1.0	1.0	59.1
	Do not know	94	24.1	24.2	83.3
	No response	54	13.8	13.9	97.2
	Not applicable	11	2.8	2.8	100.0
	Total	389	99.7	100.0	
Missing	System	1	0.3		
Total		390	100.0		

**Table 13:** Assessment of taking the HPV vaccine by respondents.

Have you ever taken HPV vaccine yourself					
		Frequency	Percent	Valid percent	Cumulative percent
Valid	No	341	87.4	87.7	87.7
	Yes	12	3.1	3.1	90.7
	No response	34	8.7	8.7	99.5
	Not applicable	2	0.5	0.5	100.0
	Total	389	99.7	100.0	
Missing	System	1	0.3		
Total		390	100.0		

**Table 14:** The assessment of either any family member of the respondents has taken the vaccine.

Has anyone in your family taken an HPV vaccine					
		Frequency	Percent	Valid percent	Cumulative percent
Valid	No	269	69.0	69.2	69.2
	Yes	43	11.0	11.1	80.2
	Do not know	65	16.7	16.7	96.9
	No response	11	2.8	2.8	99.7
	Not applicable	1	0.3	0.3	100.0
	Total	389	99.7	100.0	
Missing	System	1	0.3		
Total		390	100.0		

**Table 15:** Family member has taken the vaccine assessment.

Q207 sources					
		Frequency	Percent	Valid percent	Cumulative percent
Valid		369	94.6	94.6	94.6
	Cousin	1	0.3	0.3	94.9
	Daughter	7	1.8	1.8	96.7
	Niece	3	0.8	0.8	97.4
	Sister	3	0.8	0.8	98.2
	Sister	1	0.3	0.3	98.5
	Sister and the mother	1	0.3	0.3	98.7
	Sisters	2	0.5	0.5	99.2
	Wife	1	0.3	0.3	99.5
	Wife and daughters	2	0.5	0.5	100.0
	Total	390	100.0	100.0	

**Table 16:** Assessment of respondents' daughter is even having HPV.

Has your daughter had an HPV vaccine					
		Frequency	Percent	Valid percent	Cumulative percent
Valid	No	142	36.4	36.5	36.5
	Yes	19	4.9	4.9	41.4
	Do not know	28	7.2	7.2	48.6
	No response	32	8.2	8.2	56.8
	Not applicable	168	43.1	43.2	100.0
	Total	389	99.7	100.0	
Missing	System	1	0.3		
Total		390	100.0		

## Data Availability

The data used to support the findings of this study are included within the article.
